# Curcumin Protects against Renal Ischemia/Reperfusion Injury by Regulating Oxidative Stress and Inflammatory Response

**DOI:** 10.1155/2021/8490772

**Published:** 2021-11-13

**Authors:** Xiaoying Cui, Lili Lin, Xiaoling Sun, Lin Wang, Rong Shen

**Affiliations:** ^1^Department of Anesthesiology, The Cancer Hospital of the University of Chinese Academy of Sciences (Zhejiang Cancer Hospital), Institute of Basic Medicine and Cancer (IBMC), Chinese Academy of Sciences, Hangzhou 310022, China; ^2^Department of Anesthesiology, Qingdao Eighth People's Hospital, Qingdao 266100, China; ^3^Department of Acupuncture, Affiliated Qingdao Central Hospital, Qingdao University, Qingdao 266000, China; ^4^Department of Anesthesiology, Rizhao Central Hospital, Rizhao 276800, China; ^5^Department of Anesthesiology, Qingdao Women and Children's Hospital, Qingdao 266000, China

## Abstract

**Objective:**

The aim of this study was to explore the pharmacological effects of curcumin on oxidative stress and inflammatory response of renal dysfunction induced by renal ischemia/reperfusion (RIRI).

**Methods:**

Fifty male SD rats (Sprague Dawley) were randomly divided into the sham group, RIRI group, and curcumin group (low, medium, and high). The RIRI model was established by clipping the left renal artery for 45 min and then reperfusion for 24 h and resection of the contralateral kidney. In the curcumin group, curcumin was intraperitoneally injected once a day for 3 consecutive days using different dosage regimens. The RIRI group was intraperitoneally administered with normal saline. Renal injury was evaluated by measuring the concentration of creatinine (Cr) and urea nitrogen (BUN) in serum. Oxidative stress was assessed by assessing the level of malondialdehyde (MDA), superoxide dismutase (SOD), catalase (CAT), glutathione peroxidase (GPx), glutathione (GSH), and iron reduction/antioxidant capacity (FRAP) in tissues. In addition, the protective effect of RIRI was investigated by measuring Paller scores, the level of serum inflammatory factors and caspase-3, and the number of apoptotic cells.

**Results:**

Ischemia/reperfusion resulted in increased levels of Cr and BUN in serum and MDA in tissues and decreased levels of SOD, CAT, GPx, GSH, and FRAP. Curcumin pretreatment strikingly increased the level of SOD, CAT, GPx, GSH, IL-10, IFN-*γ*, and FRAP and significantly decreased MDA, Cr, BUN, IL-8, TNF-*α*, IL-6, and myeloperoxidase (MPO) expressions in tissues.

**Conclusion:**

Curcumin can relieve the degree of renal injury and improve renal function in ischemia-reperfusion, which may be related to the fact that curcumin can increase SOD content in serum and reduce MDA and FRAP levels in the rat model.

## 1. Introduction

Renal ischemia-reperfusion injury (RIRI) is a common clinical pathological phenomenon, which is commonly seen in vascular surgery and kidney transplantation, and is one of the common causes of acute renal failure [1, 2]. RIRI refers to that after the restoration of blood and oxygen supply to the renal organ after ischemia, the damage of the renal organ is aggravated or even irreversible, usually caused by an inflammatory cascade reaction, including reactive oxygen species (ROS), reactive nitrogen species (RNS), and cytokine, chemokine, and leukocyte activation [3, 4]. RIRI is a very complex pathological process, which mainly causes kidney damage through mitochondrial damage, inflammation, apoptosis, and oxidative stress. As an endocrine organ, the kidney is also a hyperperfusion organ, which is particularly sensitive to ischemia and reperfusion. When renal ischemia-reperfusion occurs, a large number of reactive oxygen species will be produced in the late stage of ischemia-reperfusion, which puts the kidney in a state of high oxidative stress and triggers a series of harmful cellular reactions, leading to inflammatory responses, cell apoptosis, and acute renal failure and even damage to other organs [5, 6].

Curcumin is a pigment extracted from turmeric, which is mainly distributed in tropical and subtropical areas such as India, China, and Southeast Asia. It is widely used as food pigment and has good safety in human body. Curcumin can reduce renal injury caused by renal ischemia-reperfusion by reducing oxidative stress response, upregulating APPL1 expression, inhibiting the Akt phosphorylation pathway, inhibiting activation of the INOS/NO/CGMP/PKG signaling pathway, inhibiting inflammatory cell infiltration, upregulating HO-1, inhibiting NF-*κ*B activity, and reducing the production of vasoactive substances [7, 8]. Curcumin has anti-inflammatory, antioxidant, antifibrosis, anticoagulation, and antitumor activities [9–12]. For instance, Nguyen-Ngo C et al. reported that curcumin markedly inhibited TNF-induced chemokines (CCL2-4, CXCL1, CXCL5, and CXCL8) expression, proinflammatory cytokines (IL-1*α*, IL-1*β*, and IL-6), and upregulated anti-inflammatory cytokines (IL-4 and IL-13) mRNA expression in visceral adipose tissue, human placenta, and subcutaneous adipose tissue [13]. Therefore, curcumin can be used as a new treatment method for renal ischemia-reperfusion (I/R). The purpose of this study was to investigate the protective effect of curcumin in antioxidant stress and inflammation in rats with IRI.

## 2. Materials and Methods

### 2.1. Animals

SPF male SD rats, weighing 240 ± 20 g, were provided by the Experimental Animal Center of the Nanjing University of Chinese Medicine. All experiments in this study were authorized by the Institutional Animal Care and Use Committee. SD rats were raised under standard SPF conditions, kept under controlled temperature conditions (22–24°C), dark/light cycle for 12 hours, and allowed to eat and drink freely.

### 2.2. Drugs and Reagents

Curcumin (specification: 100 g/box, lot no.: 20181209) was purchased from Bio Basic, Canada. Superoxide dismutase (SOD) and malondialdehyde (MDA) detection kits were purchased from Sigma-Aldrich (St. Louis, MO, USA).

### 2.3. Establishment of Animal Models of Ischemia and Reperfusion

After ether anesthesia [14, 15], the body temperature was maintained at 37°C, and abdominal incision through midline was performed with electrocautery to fully explore bilateral renal arteries and veins. At the same time, the renal arteries and veins were clamped bilaterally for 45 minutes. Once the ischemia time was reached, the clamps were released immediately [16]. At the end of the ischemia, the surgical area was sutured, and the rats were injected with curcumin or normal saline (NS) through a tail vein and free to get food and water. All tools used in this procedure are sterilized by autoclave or Deconex.

Throughout the procedure, a rectal probe was applied to measure the animal's temperature. A heating lamp and a heating plate were performed to keep the animal's body temperature within the range of 37 ± 1°C [17].

### 2.4. Grouping and Administration

The rats were randomly divided into 5 groups (10 in each group): sham group (Sham), renal ischemia-reperfusion injury group (RIRI), RIRI-curcumin high-dose group (60 mg/kg), RIRI-curcumin medium-dose group (30 mg/kg), and RIRI-curcumin low-dose group (15 mg/kg). The sham group and RIRI group were given the same amount of normal saline in the tail vein, and in the curcumin group, curcumin was injected into the tail vein according to the dose, for a total of 5 days [18].

### 2.5. Renal Function Assessment

After 24 h of reperfusion, rats were anesthetized with 3% pentobarbital sodium (50 mg/kg) to obtain 2–5 mL of inferior venous blood. Then, the inferior venous blood was centrifuged at 2–8°C for 10 min at 3000 rpm. Then, the upper serum was collected and stored in a refrigerator at −80°C for later experimental detection. The serum of rats was measured by an automatic analyzer (Technicon, RA-1000, USA) to evaluate renal function.

### 2.6. Renal Histomorphological Changes and Scoring

The renal tissues were fixed with 40 g/L neutral paraformaldehyde solution for 24 h, embedded in paraffin, stained with hematoxylin-eosin (H&E), and observed under a microscope: 10 fields were randomly selected, 10 renal tubules were scored in each field, and the cortical medulla was divided in half. Renal tubules were scored according to Paller criteria: 100 renal tubules were scored with a total score of 1000 points. The higher the score was, the more serious the degree of renal tubule injury was.

### 2.7. Detection of Oxidative Stress Indicators

An appropriate amount of renal tissue was taken to prepare a 0.9% renal tissue homogenate using a tissue homogenizer and then centrifuged at 3000 rpm at 4°C for 15 min to obtain the supernatant. MDA content was detected by the thiobarbituric acid method, and the content of SOD was detected by xanthine oxidase according to the instructions of the kit strictly. A total of 50 *μ*L tissue homogenate supernatant and FRAP concentration detection reagent were added to each test tube. FRAP levels were determined by measuring light absorption at 593 nm. The levels of SOD, CAT, GPX, and GSH in serum were measured using ELISA kits as per manufacturer's instructions. All reagents were purchased from Sigma-Aldrich.

### 2.8. Detection of TNF-*α*, IL-6, and IL-8 Levels

Total RNA was isolated from the entire kidney tissue using TRIzol (Japan, Takara) as per the manufacturer's instructions. Total RNA was then reversed using Advantage® RT-for-PCR Kit (Takara, Japan). Real-time PCR amplification was achieved using an ABI 7500 system (Massachusetts Thermoelectric, USA). Primers used for reverse transcription polymerase chain reaction (Invitrogen, Carlsbad, CA) are given in Table 1. Reverse transcription was performed at 95°C for 30 s and circulated at 95°C for 40 s, then at 60°C for 34 s, and then at 95°C for 15 s.

### 2.9. Determination of TNF-*α* IL-6, IL-10, IFN-*γ*, and MPO Levels in Serum

The levels of TNF-*α*, IL-6, IL-10, IFN-*γ* and MPO were detected by ELISA kit in strict accordance with kit operation instructions. All reagents were purchased from Sigma-Aldrich.

### 2.10. Statistical Analysis

Data were shown as mean ± SD. Comparisons between groups of all measured parameters were performed using the one-way ANOVA test and *t*-test. All data were analyzed using SPSS 18 statistical software. *P* < 0.05 was considered statistically significant.

## 3. Results

### 3.1. Effect of Curcumin on Renal Dysfunction

The level of Cr and BUN was strikingly increased in the RIRI group compared with sham operation (*P* < 0.01) (Figure 1(a)). In this study, significant differences in serum Cr concentrations were observed in the groups treated with different doses of curcumin during a 24-hour reperfusion period compared with the Sham group, and curcumin significantly reduced the concentration of serum Cr (Figure 1(a)). In summary, the level of serum Cr in the RIRI group was higher than those in the sham group (*P* < 0.01), while the concentration of serum Cr in the high-dose curcumin group was dramatically lower than that in the RIRI group (*P* < 0.05).

As shown in Figure 1(b), the concentration of serum BUN was 19.2 ± 1.91 mg/dL in the sham group and 58.24 ± 5.46 mg/dL in the RIRI group (*P* < 0.01). Compared with the RIRI group, curcumin at three different doses resulted in a notably lower concentration of serum BUN (*P* < 0.01); in addition, the high-dose curcumin group led to a lower concentration of serum BUN compared with medium and low doses (*P* < 0.05). The above results showed that curcumin pretreatment could reduce renal ischemia-reperfusion injury in rats, and the higher the concentration of curcumin, the more obvious the antiinjury effect.

#### 3.1.1. Renal Histopathological Observation and Score

Severe congestion and edema were observed in the renal cortex and medulla pallor in the ischemia-reperfusion group. The medulla of the curcumin group showed mild congestion and edema, while no abnormality was observed in the sham group. Under the light microscope, the renal tubules in the ischemia-reperfusion group were notably dilated, the epithelial cells were swollen, vacuolated, and granular degeneration, the capillaries in the glomerulus were dilated, red blood cells were exudated, and interstitial edema and inflammatory cell infiltration were observed. Compared with the RIRI group, the lesion of the curcumin group was prominently reduced, and the renal tissue structure of the sham group was normal. Paller scores were prominently higher in the RIRI group than in the sham group (*P* < 0.01). Paller scores of the curcumin group were prominently decreased compared with the RIRI group (*P* < 0.01), as given in Table 2.

### 3.2. Assessment of Oxidative Stress

Oxidative stress was assessed by measuring MDA, SOD, CAT, GPX, and GSH, which are the end products of lipid peroxidation caused by reactive oxygen species.  Figure 2(a) shows that the level of MDA in the sham group was 56.96 ± 4.62 nmol/kg. Compared with the RIRI group, the MDA level in the sham group was prominently increased by 78% (*P* < 0.01). Compared with the RIRI group, curcumin markedly reduced the level of MDA in renal tissues (*P* < 0.05), but still higher than that of the sham operation group (*P* < 0.01), indicating that the expression level of MDA in the curcumin group was negatively correlated with the dose of curcumin; the higher the intervention concentration of curcumin, the lower the level of MDA. The levels of SOD, CAT, GPx, and GSH in the RIRI group were 186.34 ± 8.04 U/g, 194.31 ± 11.47 U/g, 41.94 ± 3.59 U/g, and 24.97 ± 4.74 nmol/g, respectively, and markedly lower than that in the sham group (734.98 ± 12.97 U/g, 1021.73 ± 20.03 U/g, 342.94 ± 12.05 U/g, and 83.43 ± 6.03 nmol/g, respectively) (*P* < 0.05). The expression levels of SOD, CAT, GPx, and GSH in the curcumin group were markedly higher than those in the RIRI group in dose-dependent manner (*P* < 0.05), indicating that the higher the intervention concentration of curcumin was, the higher the expression level was, as shown in Figure 2. The experimental results revealed that the ischemia-reperfusion injury can produce oxidative stress in rat kidneys, and the antioxidant activity of curcumin could prevent a series of oxidative reactions. Our results also suggested that RIRI caused a significant reduction of FRAP in renal tissue compared to the sham group (*P* < 0.01). Although three different doses of curcumin increased FRAP levels, this change was only significant in the high-dose curcumin group compared with the RIRI group (*P* < 0.05).

### 3.3. Effect of Curcumin on TNF-*α*, IL-6, and IL-8 mRNA Level

As given in Table 3, TNF-*α*, IL-6, and IL-8 mRNA levels in the RIRI group were markedly higher than those in the sham group (*P* < 0.05). However, curcumin pretreatment dramatically reduced the levels of TNF-*α* and IL-8 than the RIRI group (*P* < 0.05).

### 3.4. Effects of Curcumin on Anti-Inflammatory Effects

The contents of TNF-*α*, IL-6, IL-10, IFN-*γ*, and MPO in serum of the RIRI group were dramatically higher than those of the sham group (*P* < 0.05). The expression level of IL-10 in serum of the curcumin group was dramatically higher in a dose-dependent manner than that of the RIRI group (*P* < 0.05); the higher the intervention concentration of curcumin, the higher the expression level of IL-10. The expression levels of TNF-*α*, IFN-*γ*, IL-6, and MPO in the curcumin group were memorably lower than those in the RIRI group (*P* < 0.05), indicating that curcumin pretreatment decreased the secretion of TNF-*α*, IFN-*γ*, IL-6, and MPO (Figure 3), and the expression levels of TNF-*α*, IFN-*γ*, IL-6, and MPO in the curcumin group were negatively correlated with the dose of curcumin; the higher the intervention concentration of curcumin was, the lower the expression level was, as shown in Figure 3. The results indicated that ischemia-reperfusion injury could lead to inflammatory injury of renal tissue, and the anti-inflammatory effect of curcumin could prevent this pathological process.

### 3.5. Effects of Curcumin against Apoptosis

The apoptosis number of the RIRI group was 18.87 ± 1.94, which was memorably higher than that of the sham group (7.72 ± 2.15) (*P* < 0.05). The number of apoptotic cells in the curcumin group was memorably lower than that in the RIRI group (*P* < 0.05), suggesting that the apoptosis number of cells in the curcumin group was negatively correlated with the dose of curcumin; the higher the intervention concentration of curcumin, the fewer apoptotic cells. The expression level of caspase-3 in the RIRI group was 61.96 ± 8.69 ng/g, which was memorably higher than that in the sham group (15.27 ± 2.48 ng/g) (*P* < 0.05). The expression level of caspase-3 in the curcumin group was observably lower than that in the RIRI group (*P* < 0.05), indicating that the expression level of caspase-3 in the curcumin group was negatively correlated with the dose of curcumin; the higher the intervention concentration of curcumin, the lower the expression level, as shown in Figure 4. The results showed that curcumin alleviated renal ischemia-reperfusion injury via exerting the antiapoptosis effect.

## 4. Discussion

Ischemia-reperfusion injury leads to the deterioration of the function of the transplanted kidney after the restoration of blood supply [19]. RIRI is the main cause of acute kidney injury after partial nephrectomy and kidney transplantation [20], which is closely related to morbidity and mortality [21]. Therefore, effective preventive and therapeutic measures are necessary to reduce renal ischemia-reperfusion injury. Inflammation is an important pathophysiological mechanism of RIRI. RIRI can induce inflammatory cell aggregation, release inflammatory factors (such as TNF-*α*, IL-6 and IL-8), and increase adhesion molecules, which together stimulate inflammatory cascade, leading to organ damage [22]. After renal ischemia, renal cell ischemic necrosis occurs, and then, restored perfusion can cause secondary damage to the kidney [23]. When renal function injury reaches a certain degree, it can exacerbate the level of BUN and Cr [5].

Current studies on the prevention and treatment of RIRI mainly focus on antioxidants and antiapoptotic drugs [24]. Curcumin is an extract from the rhizome of turmeric, which is an orange knot powder and is widely used as pigment, food additive, and condiment [25]. Previous studies have shown that curcumin has antioxidant [26], anti-inflammatory [27], immunomodulatory [28], and antimicrobial effects [29]. At the same time, curcumin has little toxic and side effects in rodents and humans, and no obvious adverse reactions have been observed even at high doses [30]. Therefore, curcumin has broad medicinal prospects.

The results of this study showed that serum Cr and UBN were highly elevated in the RIRI group, possibly due to a sharp decrease in glomerular filtration rate (GFR) and significant damage to renal tubule function in the RIRI group, and the application of curcumin resulted in partial recovery of renal function and reduced oxidative stress induced by RIRI. The content of BUN and Cr in the RIRI group was higher than those in the sham group, indicating that renal function was obviously damaged. After curcumin treatment, serum BUN and Cr decreased signally, indicating that curcumin has a protective effect on renal function, which is consistent with the findings reported in the literature [6].

When RIRI occurs, the mitochondria of kidney cells are also damaged, leading to decreased activities of SOD and GSH and being unable to effectively remove oxygen free radicals in the body, resulting in the disorder of the body's redox system and aggravating body damage. Curcumin has antioxidant effects and can regulate the activities of GSR, CAT, and SOD in free radicals, thus playing an antiinjury role. Endothelial cell dysfunction during RIRI can produce many inflammatory mediators and release a variety of inflammatory transmitters and adhesion molecules, leading chemotactic neutrophils and inflammatory cells to adhere to vascular endothelial or enter cells. At the same time, neutrophils and other inflammatory cells themselves can release chemotactic substances, which act on the kidney and cause renal ischemia-reperfusion, further aggravating kidney injury. In our study, ischemia/reperfusion resulted in an increased level of MDA and a reduced level of FRAP in the renal tissues of the RIRI group, which was consistent with the previous studies [31]. The content of SOD in the RIRI group was lower than that in the sham group, while the content of MDA was higher than that in the sham group, indicating that after renal ischemia and reperfusion, the body showed obvious lipid peroxidation reaction and weakened antioxidant capacity. Compared with the RIRI group, the content of SOD significantly increased and the content of MDA decreased in the curcumin group, indicating that curcumin treatment can reduce the content of oxygen free radical and inhibit biofilm lipid peroxidation caused by oxygen free radical accumulation, thus enhancing the antioxidant capacity of the kidney and protecting renal ischemia-reperfusion injury [32].

The limitation of this study is that there is no further study on the downstream signaling pathway in which curcumin plays a role. In future studies, we will apply fluorescently labeled curcumin to explore the way in which it acts on cells, such as cell surface receptors or endocytosis.

In summary, curcumin plays a protective role in renal function by preventing cell damage and inhibiting cellular oxidative stress, inflammatory response, and apoptosis, but the specific protective and repair mechanism needs further exploration.

## Figures and Tables

**Figure 1:** (a) The concentration of serum Cr in rats in the RIRI group, sham group, curcumin group L, M, and H, and renal ischemia-reperfusion group. (b) The concentration of serum BUN in rats in the RIRI group, sham group, curcumin group L, M, and H, and renal ischemia-reperfusion group (^∗∗∗^*P* < 0.01, vs. the sham group. ^#^*P* < 0.05, vs. the RIRI group). L, low; M, medium; H, high.

**Figure 2:** Protective effect of curcumin on ischemia-reperfusion injury in rats. The levels of MDA (a), SOD (b), CAT (c), GPX (d), GSH (e), and FRAP (f) in renal tissues are detected. ^∗^*P* < 0.05, vs. the sham group. ^#^*P* < 0.05, vs. the RIRI group.

**Figure 3:** Effect of curcumin pretreatment on expression of TNF-*α*, IFN-*γ*, IL-6, IL-10, and MPO in the kidney after renal ischemia-reperfusion injury.

**Figure 4:** Effect of curcumin pretreatment on apoptosis of ischemia-reperfusion injury rats vs. the sham group, ^#^*P* < 0.05, and vs. the RIRI group, ^∗^*P* < 0.05.

**Table 1:** Real-time quantitative PCR primer.

Gene	Sense strand sequence	Antisense strand sequence
TNF-*α*	AACACGAGTGACAAGCCCGTAG	GTATCACCAGTTGGTTCTCTTTGA
IL-6	AGGTTCCATGTGCAAGTGTCT	GACAGCCCTGGTCAAAGGTT
IL-8	CTGCAAGAGACTTCCATCCAG	AGTGGTATAGACAGGTCTGTTGG
*β*-Actin	AGAGGGAAATCGTGCGTGAC	CAATAGTGATGACCTGGCCGT

**Table 2:** Comparison of Paller scores in rats.

Group	*n*	Paller score
Sham group	10	103.29 ± 16.38
RIRI group	10	509.23 ± 30.07
Low-dose curcumin group	10	430.97 ± 25.13
Medium-dose curcumin group	10	397.58 ± 20.75
High-dose curcumin group	10	351.34 ± 17.59

**Table 3:** Effects of curcumin pretreatment on TNF-*α*, IL-6, and IL-8 mRNA levels in the kidney after renal ischemia-reperfusion injury.

Group	TNF-*α* (mRNA)	IL-6 (mRNA)	IL-8 (mRNA)
Sham group	1.07 ± 0.19^∗∗^	1.14 ± 0.21^∗∗^	0.96 ± 0.118^∗∗^
RIRI group	12.36 ± 1.85	5.09 ± 0.37	7.63 ± 0.82
Low-dose curcumin group	6.53 ± 0.99^∗^	2.07 ± 0.52^∗^	3.77 ± 0.46^∗^
Medium-dose curcumin group	5.87 ± 0.43^∗^	1.76 ± 0.47^∗^	2.49 ± 0.38^∗^
High-dose curcumin group	4.74 ± 0.34^∗^	1.48 ± 0.39^∗^	2.01 ± 0.17^∗^

^∗^ *P* < 0.05, ^∗∗^*P* < 0.01, vs. the RIRI group.

## Data Availability

The data used to support the findings of this study are available from the corresponding author upon request.
